# An Empirical Analysis of the Role of Piano Performance in Alleviating Psychological Trauma in People with Psychological Isolation Disorder

**DOI:** 10.1155/2022/4024852

**Published:** 2022-06-11

**Authors:** Xia Cao

**Affiliations:** College of Music, Shanxi Normal University, Linfen City, 041004 Shanxi Province, China

## Abstract

This paper presents an in-depth analysis and study of the role of piano performance in alleviating psychological trauma in people with psychological isolation disorder. In this paper, we designed a music modulation system based on EEG signals of people with isolation disorder and designed an interface with real-time emotion recognition. MATLAB is responsible for data processing and classification, while Python is responsible for communication and real-time transmission between modules, EEG signal collection, and processing. For the EEG signals in the DEAP emotion database, a Butterworth bandpass filter is used to denoise the signals, and then, a wavelet packet decomposition reconstruction is used to remove the artifacts and complete the preprocessing of the signals. Finally, the support vector machine with optimized parameters of the genetic algorithm was used to classify the positive, neutral, and negative samples with 89.23% accuracy. In this study, all subjects were divided into experimental and control groups by experimentally measuring the changes in heart rate, skin electrical conduction, skin temperature, and EEG signals before and after the experimental group, and statistical analysis was also performed on the data tabulation of the experimental and control groups. The experimental results proved that piano playing has a significant effect on relieving the psychological trauma of people with psychological isolation disorder when the training frequency of piano playing therapy reaches a certain intensity. This study provides a certain theoretical basis for clinical, educational, and health services.

## 1. Introduction

Music is a kind of art, the sound is born from the heart, and it is the product of people's mental activity. Music not only has a certain appreciation and aesthetic value but also has a certain therapeutic effect. Music therapy is a new and emerging interdisciplinary discipline that integrates music, medicine, and psychology, which is the application and development of the role of music outside the traditional art appreciation and aesthetic field [1]. Music is a magical thing, with a unique charm. Human ancestors used songs to warn of imminent danger, to share the joy of success, to vent their anger, and to help a person vent his or her inner emotions (McDermott O, 2018). It is because music is so richly expressive that its effects are impressed upon the human brain to the fullest [2]. Historical practice shows that music occupies an important place in the life of the whole society because it transcends language and facilitates communication between people. In the process of enjoying music, musical information (including rhythm, melody, harmony, and timbre) plays a good role in facilitating the overall function of the brain, which is manifested as enhanced memory and active thinking. Music can also induce the potential great power in people's hearts, make the mind many scattered and isolated information from each other combined, and promote the development of creative thinking [3].

Situational emotional understanding plays an important role in normal social interactions for individuals with autism. In daily life, social interaction with others is essential to recognize the emotions of others, but recognizing the emotions of others can be based not only on their facial expressions but also on certain contextual cues, which is a form of contextual emotion understanding [4]. Studies have shown that individuals with autism have deficits in facial expression recognition, but is this still true for contextual emotion understanding? As a special population with pitch perception and a certain ability to recognize musical emotions, can music help individuals with autism to activate their emotion recognition? Both music and context can express emotions, so theoretically, children with autism could also activate the activation of contextual pictures through the recognition of musical emotions. Also, there are relevant empirical studies that show that musical emotions can influence the recognition of emotional words and faces in normal people [5]. Therefore, further research is necessary on emotion activation experiments with withdrawn children. Investigating whether music can be used to enhance the recognition of contextual emotions in children with autism will contribute to the development of music therapy interventions.

Since the 1960s, the prevalence of withdrawn children has continued to rise, and according to the Centers for Disease Control and Prevention, the prevalence of withdrawal disorders has reached 1 : 69 in 2018, with U.S. researchers finding that there is an estimated 1 in 45 children with withdrawn disorders in their surveys. An increasingly prominent issue for children with autism is “social communication and social interaction,” which manifests as emotional and behavioral difficulties and inappropriate behavior, and without addressing this issue, other rehabilitation and education for children with autism are difficult. For example, a child with autism may suddenly cry in class and hit his or her head, leap from his or her seat and run around wildly, or even hurt others. For this reason, this study tries to investigate how to alleviate the psychological trauma and improve the emotional behaviors of the withdrawn people through piano playing, to make these people better interact with others in the integrated education environment and daily life, against the background of such a high prevalence of withdrawnness.

## 2. Related Works

Research on music therapy began in the United States in the early 20th century, with music therapy being used early on for patients with significant physical and mental impairments and gradually expanding after World War II to include treatment for children and adults with special needs affected by intellectual, physical health, mental health, and participation in social activities (such as soldiers in World War II) [6]. Some American researchers have described music therapy as a systematic intervention process in which the music therapist interacts with the patient in different types of musical experiences to achieve therapeutic goals. Dr. Nagel of Japan has given another interpretation of music therapy in the context of his profession, arguing that music is medicine for the music therapist as a physician [7]. The doctor uses music as a medium to prescribe different types of prescriptions and treats the patient together through the assistance of music therapists, music creators, nurses, psychologists, and other members. Music therapy involves the elicitation of the emotions of the withdrawn child and the switching of music to regulate and guide the emotional state of the withdrawn child so that his or her emotions eventually stabilize. For example, Koelsch conducted an experiment to induce different emotional states in the subjects, and the subjects' emotions of joy, anger, and sadness were induced by different types of audios, and the classification and identification of emotions were accomplished by recording and analyzing their EEG signals and extracting the features in the EEG signals. Music therapy can combine music and pictures to induce emotions from both auditory and visual dimensions [8]. Weber, an American scholar, designed and developed pictures showing six emotions: happiness, anger, sadness, surprise, disgust, and fear as visual evocation sources, and the series of pictures were widely used by researchers, who combined emotional pictures with their corresponding audio materials to conduct experiments [9]. The independent sample *t*-test was used to detect whether there were differences between the two groups in factors such as age and intelligence, the exact probability method was used for demographic data analysis, and groups (experimental group, control group) were used as between-subject factors, and emotional consistency (emotional consistency, emotional inconsistency) was a repeated-measures analysis of variance (ANOVA) for the subject's situational emotion and musical emotion recognition ability as a within-subject factor.

Regarding the research on the emotional behavior of children with autism, some people have started from the medical level to empirically prove the effectiveness of music therapy on the emotional behavior intervention of children with autism, such as Kasl-Godley, who closely integrated physiology and music therapy in clinical practice and found that rhythms occur between music's own regular sound wave vibration frequency and internal resonance, which will regulate the reticular structure of the brain through music, making the limbic system TEM, cerebral cortex [10]. Ribeiro discovered the EEG mechanism of music on emotion by exploring the association between music and emotion [11]. Unbehaun selected 40 cases of autistic children admitted to the hospital for music therapy and found that it could significantly improve the perceptual and behavioral abilities of the children and improve their emotions [12]. For example, Knott used 30 cases of children with autism, 22 aged 1-3 years and 8 aged 3-7 years, applied the passive listening method, active participation method, improvisation method, and suggestive relaxation method in music therapy to statistically analyze the emotional-emotional interactions and behavioral development before and after the treatment, and found that the developmental level after the treatment was higher than before the treatment, mobilized [13]. It was found that the treatment resulted in higher levels of development than before the treatment, mobilization of positive emotions and reduction of stereotyped behaviors, as well as longer attention span, wider attention span, increased eye contact, and improved verbal expression. Skin conductance level is often used as an indicator of emotional intensity, and an increase in skin conductance level indicates enhanced emotional activity.

Because of the rapid growth of the population with autism and the urgent need for rehabilitation of the autistic population, research efforts are being accelerated both in Japan and abroad. According to the existing situation in foreign countries, the understanding and research on the autistic group are relatively mature, and the construction of barrier-free facilities in the public environment is well developed. For the domestic situation, with the continuous improvement of social civilization and the rapid development of the economy and technology, the government and the society pay more attention to the educational rehabilitation and medical rehabilitation of disabled people, and the facility rehabilitation plays a pivotal role in the support services for disabled people as a part of the support system for disabled people's service security [14]. At the same time, to carry out better rehabilitation services in the future, we need the government's legislative and other policy support. We should strengthen the legislative work of the National and Local People's Congresses for the rehabilitation of people with disabilities and establish a perfect legal system, which is conducive to the organizations of the Disabled Persons' Federation to explicitly include the education and training of autistic groups into the scope of work, start to formulate specific policies and carry out practical work, assist in the promotion and popularization of knowledge about autism, and organize relevantly. We will also help to promote and popularize the knowledge of autism, organize training for professionals, and so on, to effectively protect the fundamental interests of the autistic group. In this study, heart rhythm, skin temperature, and skin electrical conduction level were selected as indicators, and it was found that during the treatment process, all three were changed.

## 3. Design of a Trauma Model Based on Piano Performance to Alleviate the Psychological Isolation Disorder Population

In terms of average reaction time, the reaction time of the experimental group was slower than that of the control group whether it was emotionally consistent or emotionally inconsistent. People with withdrawn disorders often wander into their closed behavioral systems due to fear of injury. When there is a sense of dependence on some things, the attention to other things will be drastically reduced. Therefore, it is important to try to exercise them to break their unchanging system by putting the thing they focus on in a different position each time, changing the color, and so on, to make their system more flexible. As shown in Figure 1, the change in the peripheral system is the intervention in which the horizontal dimension occurs, and the peripheral system, the behavioral system, of the withdrawn child both are the measures in which the vertical dimension intervention occurs [15]. In general, the “person,” who is often present in the peripheral system, influences the change in the relationship in a dominant way. In what way do the “person” and the peripheral system, the behavioral system of the withdrawn child, change? In real life, we can imagine a vehicle that allows the behavior of the autistic person to be influenced by the person in the peripheral system and to influence the life of the autistic person, creating a mutual exchange between the two.

The issue of human involvement is more common in people with autism and can be considered an important part of the intervention. They are more receptive to the help and companionship of their loved ones compared to the norm, but when a stranger they do not know walks in on them, it can make them feel panicked and scared. Therefore, people and things can change throughout the process of environmental rehabilitation for people with autism. For example, if there are things that the withdrawn child likes very much, it is necessary to let them try to accept new things. The classifier needs to be pretrained before recognizing emotions, in order to find better parameters to make the classifier more accurate. The features of multiple physiological signals are fused into a joint vector, and the feature vector after dimensionality reduction of the joint vector is used as the input data of the logistic regression classifier. The present study included three experiments to explore subjects' ability to recognize musical emotions and contextual emotions. Experiment 1 was a single-channel emotion priming experiment, in which the priming stimulus and target stimulus were the same as the contextual emotion picture. Experiments 2 and 3 were cross-channel emotion priming experiments in which the priming stimulus and target stimulus were the contextual emotion picture and music stimulus pair and the music stimulus and contextual emotion picture pair, respectively. All experimental tasks were preceded by 8 practice trials, and the formal experiments contained a total of 96 trials, with 48 trials for happy and sad emotions, 48 trials for all happy and sad emotions paired as emotionally incongruent, 24 trials for happy and happy emotion stimuli paired as emotionally congruent, and 24 trials for sad and sad emotion stimuli also paired as emotionally congruent conditions.

The kernel function parameters are selected as follows: the polynomial kernel function *q* ≥ 1 is the polynomial degree; the penalty factor in the radial basis kernel function is *c* = 2, *δ* = 60; the sigmoid kernel function *v* > 0, *c* > 0.  Figure 2 shows the effects of SVM classifiers with four different kernel functions on emotion recognition based on physiological signals.

The procedure of the cross-channel emotion recognition experiment: each trial starts with a 300 ms black cross in the middle of the screen, followed by a 500 ms blank screen, followed by a 200 ms start stimulus, which is a standardized music chord with emotion. After a 50 ms interval of the blank screen, the target stimulus appeared, and the target stimulus was a standardized mood picture, and the subject needed to determine as quickly and accurately as possible whether the mood picture was happy or sad after listening to the music. After the subject responded with a keystroke, the string “XXX” appeared on the screen for a certain length of time (1000 ms or 1020 ms) as a masking stimulus, and after the masking stimulus ended, the next round of target stimuli would appear again for the subject to judge.

(1) $$\begin{array}{c} f\left(x\right)=\sin\left(\underset{i=1}{\sum }a_{i}y_{\varphi }\left(x_{i},y_{i}\right)\right). \end{array}$$

The human cerebral cortex is involved in perceptual, cognitive, and emotional activities including attention, behavior, volition, perception, reasoning, learning, and memory. The cerebral cortex is composed of tens of billions of neuronal cells and is an extremely large and complex network of neurons. The main formation of the EEG signal is formed by the sum of the postsynaptic potential changes in the parietal dendrites of the cerebral cortex cells, which are generated by the mutual transmission of neuronal network discharges. The stronger the generated electrical signal, the more intense the brain complementary activity. Potential changes of -20 to 20 mV recorded in the absence of experimental stimuli are called “noise.”

The article uses EEG data from the DEAP database, a standard multimodal affective database established by Witusik et al. in 2019, to validate the algorithm. EEG signal data were collected from a total of 40 volunteers, with a 50/50 ratio of male and female volunteers [16]. The volunteers were in good physical and mental health at the time of the experiment and had normal hearing and vision. Forty sensors were placed in four areas of the brain to collect EEG signals, and eight sensors were placed in other areas of the brain to collect voluntary physiological signals such as electrooculography (horizontal and vertical eye), electromyography (zygomatic and trapezius muscles), electrodermal, respiratory rhythm, volume changes, and body temperature. EEG and autonomic physiological signals were collected from volunteers enjoying 40 s of piano playing, with each experiment enjoying a piece of piano playing. The experiment number of the experiment was displayed for 2 s at the beginning of the experiment, followed by 5 s of the baseline score, and finally 60 s of the randomized audio emotion-evoking material, during which the physiological signals of 48 channels were recorded. After the channels were selected, the baseline drift was removed by calculating the mean value of the signals and removing the baseline signals for the first 5 s. The remaining 60 s of EEG data were preprocessed. All subjects had normal hearing or corrected hearing, each subject was healthy and had a good sleep before participating in the experiment, and there was no history of brain disease and no history of drug and alcohol abuse.

(2) $$\begin{array}{c} y=wx+b+\xi \leq 1. \end{array}$$

There is a lot of low-frequency noise in the signal, such as respiration, dermatographia, and cardiac. In this experiment, a fifth-order Butterworth bandpass filter from 1 Hz to 50 Hz was used to remove the low-frequency noise below 1 Hz. After filtering, the obvious noise signal has been removed, but there are still artifacts; the most obvious of which is the electro ocular artifacts. Because of the small number of device channels used in this experiment, if the channel in the forehead region near the eye is selected as the reference electrode for the independent component analysis method, the number of channels used for emotion identification will be reduced.

(3) $$\begin{array}{c} \log_{y+1}=\frac{x\theta^{T}-b}{1-y},\\ x\left(t\right)=\overset{N}{\underset{i=1}{\sum }}\left(a_{i}y_{\varphi }+u_{i}s_{i}\right). \end{array}$$

To calculate the BF, the competing hypotheses for population-standardized effect sizes were first specified*δ*: *H*_0_ assumes no differences between groups or conditions (*δ* = 0), while *H*_1_ assumes the presence of a true effect (*δ* ≠ 0). In Bayesian *t*-tests, the prior distribution *H*_1_ is chosen by default to be the Cauchy distribution centered at 0 with *r* = 0.713, i.e., *H*_1_ : *δ* ~ Cauchy(0, 0.713). BF_incl_ can provide evidence for or against the inclusion of an effect or interaction and is interpreted by the same strength-of-evidence threshold as BF_incl_. Bayesian four-factor ANOVA was calculated using a default parameter prior (fixed effects *r* = 0.5, random effects *r* = 1, and covariates *r* = 0.354) forBF_incl_, and the subject factors were treated as random effects. For multifactor ANOVA, *H*_1_ is defined as including a main effect or an interaction. When there was sufficient evidence of interaction (BF_incl_ > 3), a Bayesian *t*-test was conducted to compare the difference between the two levels of mood congruence and mood incongruence.

(4) $$\begin{array}{c} {\text{BF}}_{\text{incl}}=\frac{1}{N}\underset{k=1}{\sum }\left|x_{i}\left(k^{2}\right)\right|\sqrt{3},\\ w^{T}\cdot x-2b^{2}=1. \end{array}$$

Traditional null hypothesis significance tests were conducted using IBM SPSS version 22.0. Independent samples *t*-tests were used to detect the presence of differences between the two groups of subjects on factors such as age and intelligence, demographic data analysis using the exact probability method, and repeated measures ANOVAs on subjects' situational emotion and musical emotion recognition abilities using group (experimental, control) as a between-subjects factor and emotional congruence (emotional congruence, emotional incongruence) as a within-subjects factor. Pachelbel's “Canon in D major” is a representative of quiet and light tones. The soothing and gentle tune can make the listener feel happy, forget troubles and sorrows, and devote themselves to the wonderful world constructed by music. Now, when Beethoven's “Fate” sounded, the oppressed indignation gushed out, instantly evoking people's thoughts. Therefore, the choice of Canon in D major and Destiny is representative. When the original hypothesis test is not significant, that is, when it concludes that there is a significant difference or effect, but this design may not detect significant differences or the strength of the interaction. From another perspective, when the results are not significantly different, it is also not possible to distinguish whether the results are due to the absence of evidence or their inherent absence of significant differences. In this case, Bayes factors and equivalence tests provide support for the lack of a meaningful effect. The corresponding descriptive statistics for correctness and reaction time of situational emotion recognition of the withdrawn individuals were performed using SPSS 22.0 and plotted using origin version 2021, and the results of the analysis are shown in Figure 3. In terms of the average reaction time, the reaction time of the experimental group was slower than that of the control group in both the consistent and inconsistent mood conditions; in terms of the average correct rate, the correct rate of the experimental group was lower than that of the control group in both the consistent and inconsistent mood conditions.

Based on the algorithm design and validation in the previous section and the emotion model based on the EEG signal data obtained from the emotion elicitation experiment, this study designed a piano performance-based trauma mitigation system for people with psychological isolation disorder. In this section, the system is described in terms of the introduction of the system, the software design of each module of the system, and the use and functions of the GUI human-computer interaction interface, and the system is tested at the end. The system has the functions of data analysis of EEG signals, training of models, real-time recognition of emotions, and automatic switching of music material to play [17].

The music regulation system based on children with autism can monitor the emotional state of children with autism in real time when they are undergoing music therapy. The EEG signal is collected by the EEG device, and the system preprocesses feature extracts and classifies the EEG signal and displays the classification results in the system interface in real time. The system will judge whether the type of music needs to be switched according to the recognition result. When the system detects for the first time that the user's EEG signal state reaches the standard of needing to switch music, the system will switch the currently played music video material to a heterogeneous material opposite to the current emotional state, and when the system detects for the second time that the user's EEG signal state needs to switch music, the system will switch the currently played music video material to neutral. In this process, feedback is formed, the EEG device transmits the EEG signal to the system in real time, and the system continuously monitors the emotional state and controls the piano playing instructions. The system flow is shown in Figure 4.

## 4. Analysis and Discussion of the Study Results

### 4.1. Model Performance Testing

The classifier needs to be pretrained before recognizing emotions, intending to find better parameters to make the classifier more accurate. The features of multiple physiological signals are fused into a joint vector, and the joint vector is used as the input data for the logistic regression classifier after dimensionality reduction. The main parameters of logistic regression are regularization type (penalty) and *C*. There are two main types of regularization types, *L*1 and *L*2, and the value of *C* is [0.1, 1, 10, 100], which is set to prevent overfitting. In this chapter, the emotion recognition study only focuses on anxiety, pleasure, and calming emotions to do targeted work for the subsequent reconfiguration of the stress reduction music system. Logistic regression is a two-classifier model that identifies the results after the fusion of features of multichannel physiological signals, which can identify anxiety emotions and calm emotions. The partial results of classifying anxiety and calming emotions under different parameters are shown in Figure 5.

Music occupies an important position in the whole social life because it transcends language and facilitates the communication between people. Music can also induce a huge potential in people's hearts, so that many scattered and isolated information in the mind can be combined to promote the development of creative thinking. To determine the effect of kernel functions on the accuracy of classifier classification, the reduced-dimensional feature vectors were sequentially input into a support vector machine with four different kernel functions for comparison. The kernel function parameters were chosen as polynomial kernel function *q* ≥ 1 for the polynomial count; penalty factor in radial basis kernel function*c* = 2, *δ* = 60; and sigmoid kernel function *v* > 0, *c* > 0. The SVM classifiers with four different kernel functions for physiological signal-based recognition of emotional effect are shown in Figure 2.

After training the SVM classifier and the logistic regression classifier separately, the EEG, ECG, and respiratory signals were extracted and fused into a joint feature vector, which was input into the classifier after dimensionality reduction, and the two different classifiers were compared for the accuracy of emotion recognition after fusion of multichannel physiological signals. This multichannel feature-level fusion emotion recognition model uses an SVM classifier to recognize anxiety and calm emotions with an accuracy of more than 80% and logistic regression classifier to recognize the highest accuracy of 76.89%. The SVM was more accurate than the logistic regression classifier for both emotions, so the recognition model used a binary SVM classifier for emotion recognition. In this experiment, a fifth-order Butterworth bandpass filter from 1 Hz to 50 Hz is used to remove low-frequency noise below 1 Hz. After filtering, the obvious noise signal has been removed, but there are still artifacts, the most obvious of which is the electrooculography artifact.

### 4.2. Subjects' Emotional Behavior Statistics

In this study, all subjects had a normal hearing or corrected hearing, each subject was in good health and slept well before participating in the experiment, and none had a history of brain disease and no history of drug or alcohol abuse [18]. Before starting the experiment, the subjects were informed of the purpose of the experiment, the procedure, and related precautions and were told to minimize blinking and body movements during the experiment to reduce the interference of optoelectrical and electromyographic signals. At the same time, the subjects were informed that the experiment was safe so that they could relax and perform the experiment smoothly. In this experiment, a 32-channel electrode cap made by NEURACLE was used, and the international 10/20 rule was used to place the EEG signal with a sampling frequency of 1000 Hz, and a total of 32 channels of EEG signals were acquired. The four components work together to acquire EEG signals.

Subjects leaned back in a chair, wore headphones, and were about half a meter from the display laptop screen. The ambient temperature of the laboratory was 25 degrees, quiet and comfortable, and the fluorescent lights were turned off during the experiments. The experiments started at 2:00 p.m. and lasted approximately 45 minutes. The experiments were prepared for about 30 minutes by setting up the equipment and injecting conductive paste. Subjects will perform three tests, each lasting approximately 5 minutes.

Sample entropy has two advantages: sample entropy has better consistency: (1) the calculation of sample entropy does not depend on the length of the data; (2) sample entropy has better consistency; that is, changes in the parameters *m* and *r* have the same degree of impact on the sample entropy. The lower the value of the sample first, the higher the sequence self-similarity; the larger the value of the sample first, the more complex the sample sequence. C (central) denotes the central region, F (frontal) denotes the frontal region, FP (frontal pole) denotes the frontal pole, P (parietal) denotes the parietal region, T (temporal) denotes the frontal region, and O (occipital) indicates the occipital region. The numbers represent the left and right sides, odd left and even right.

Taking Pachelbel's Canon in D major and Beethoven's Fate as examples, the results of sample entropy processing showed that the sample entropy of leads was slightly higher for synchronous stimuli than for visual stimuli alone, except for frontopolar FP1 and FP2 and central parietal CP1 and CP6. Most other brain regions had lower mean audiovisual sample entropy with red video stimuli alone. The lowest sample entropy values were found for music, indicating that brain activity under a single auditory stimulus had the lowest time-series complexity and was more regular compared to visual stimuli and audiovisual year-on-year stimuli, as shown in Figure 6.

Try to put the things he focuses on in a different position each time, and change colors and other means to train them to break the original immutable system and make their system more flexible. Twenty negative stimulus pictures were selected from the Emotional Picture System CAPS. The same type of pictures was used to induce bad emotions, and the consistency of the same type of pictures in the two dimensions of validity and arousal was high so that when the pictures were switched, the state of the subjects fluctuated less and the stability of emotions could be ensured. In this way, when switching between pictures, the subjects' state fluctuates less, and the stable emotion can be ensured, which enhances the evoking effect while avoiding the monotonous content that leads to the subjects' fatigue [19]. The experiment was divided into two groups, namely, the control group and the experimental group. Each picture was displayed for 5 seconds and played continuously, and the subjects completed the experimental exercise before the experiment. EEG data were not collected to familiarize the subjects with the experimental interface and procedure. Based on the raw data of the 24 recovered emotion self-assessment forms. After processing, the results were obtained as shown in Figure 7, and it was found that after the experimental intervention, the subjects in the experimental group had significantly higher emotional self-rating values than the members of the control group.

The comparison of the self-rated values shows that the experimental group who watched the blue video had significantly higher self-rated values of “happy and relaxed” than the control group. For the control group who did not watch the blue video, the self-rated values of “fear, disgust, sadness, and anger” were higher than those of the experimental group. For neutral emotions, the difference between the two groups was not significant. The visualization of music with blue and green audiovisual stimuli was more regular than that of red, which has a certain effect on the soothing regulation of brain emotions. Autism is a pervasive brain disorder that typically appears in the first three years of childhood and persists throughout a person's life. People with autism may be more engaged in their own ideas and unable to engage in social activities; they may also have behavioral problems and language impairments (such as imitating language). People with autism often respond abnormally to sounds, perceptions, and other sensory stimuli.

By improving the psychological trauma of solitary disorder through piano playing therapy, the external symptoms are changing and there are changes in the level of internal psychological qualities. At the same time, the musical intervention was accompanied by changes in physiological indicators. In this study, heart rhythm, skin temperature, and skin electrical conduction level were selected as indicators, and all three were found to change during the treatment [17]. There were individualized differences in the characteristics of the changes. Under the piano playing intervention, the physiological indicators of the body will change. Resp rate is the indicator of heart rate change, Temp makes the indicator of skin temperature change, the decrease of skin temperature is the expression of relaxation of the body, and the increase is the expression of tension; Skin Cond indicates the skin's electrical conduction. The rise or fall of skin conductance value also reflects the relaxation and tension of the body. The galvanic skin response apparatus was first called the psychometric reflex. During emotional states, changes in vasodilation and contraction in the skin and sweat gland secretion can cause changes in skin resistance. The galvanic skin response apparatus is used to reflect the emotional response of the vegetative nervous system. The skin conductance level is often used as an indicator of emotional intensity. An increase in skin conductance level indicates increased emotional activity, such as an increase in skin conductivity and skin current when the body is fatigued. An increasingly prominent problem in children with autism is “social communication and social interaction,” which manifests as emotional behavioral disturbances and inappropriate behaviors. For example, an autistic child suddenly cried out inexplicably during class or suddenly banged his head in a frenzy. None of these behaviors can make it integrated into normal body life and education.

In the piano playing intervention condition, the overall change in heart rate fluctuations shows a regular periodicity. However, it is influenced by the feedback of the music rhythm; i.e., the heart rate fluctuations are also intensified under the effect of fast-paced music. There is a significant change in the peak heart rate when the music track is changed, as shown in Figure 8. In the figure, the horizontal coordinates indicate time and the vertical coordinates indicate heart rhythm; in the later appearing figures, the horizontal coordinates also indicate observed values reflecting changes in time, and the vertical coordinates indicate observed values reflecting changes in the corresponding physiological indicators and similarly later.

### 4.3. Effectiveness of Trauma Mitigation Strategies for Piano Performance

In this study, five of the 40 subjects were randomly selected for long-term follow-up, and the following conclusions were drawn. The number of times the subjects' emotional behaviors occurred after the intervention. The developmental graph of the number of times the subjects' emotional behaviors occurred after the intervention showed that the frequency of each of the five subjects' emotional behavior problems had decreased significantly at the beginning of the thousand preintervention, and by the maintenance period, two of the subjects' emotional behaviors had subsided and one subject's emotional behavior had also diminished to 0-1 times per week. As shown in Figure 9, the horizontal axis indicates the number of weeks of the experiment and the vertical axis indicates the subjects' emotional behaviors occurred.

As a special population, autism has pitch perception and a certain ability to recognize musical emotions. The treatment plan based on music therapy for autism emerges as the times require. The Parent Interview Form (post 1000 pretests) and the Teacher Interview Form (post 1000 pretests) captured a significant increase in subjects' self-control and a significant increase in the duration of listening eye contact and verbal interaction. The researcher used the Parent Interview Form (postintervention) and the Teacher Interview Form (postintervention) to interview the parents and teachers of the five subjects again at the end of the experiment, and the results distilled from the interview data showed that several interviewees unanimously indicated that the subjects' emotional behavior state after the music therapy training completely exceeded their envisioned expectations and considered the music therapy program to be very effective and of great importance, socially significant and worthy of replication for withdrawn children with severe emotional behaviors. Parents and classroom teachers agreed that the piano playing in this study subdued or attenuated the emotional behaviors of the withdrawn children and had a transfer and generalization effect with the help of parents and teachers, which had a very good impact on the children's learning and life, as well as on family interaction and classroom order. These directly indicate the good social validity of this study.

## 5. Discussion

In the past two decades, people have been paying increased attention to special education, and the methods and measures of special education have been gradually improved, but at present, the target of international special education is mainly children with disabilities, and the attention and help given to children with special needs like autistic children are much less than those with disabilities. More attention needs to be paid to future teaching and research. At the same time, the government should also give strong support in terms of measures and related facilities and equipment and strictly examine the qualifications of treatment institutions to help people with psychological autism integrate into normal group life as soon as possible. At the same time, the parents of people with autism should also formally recognize the disease and actively cooperate with the treatment. In the eyes of many parents, it is difficult for them to accept other people saying that their child has such a disorder out of love for them. So, when others remind parents that their child is not capable in a certain way and needs to be taken seriously, they find various reasons to refute this, such as the fact that each child grows differently, that a 2-year-old child does not respond to anyone calling his or her name, that he or she is serious about something, and so on. Because they do not want to accept that their child is lagging behind other children, they do not take these phenomena seriously and treat them as diseases.

The analysis of the above assessment form as well as the interview of learning outcomes and the observation of teaching outcomes revealed that Xiao Xi, a child with high-functioning autism, enjoyed piano learning by being exposed to piano playing as an experiment. This skill of piano learning greatly improved his physical coordination, especially his fine motor skills. In addition, he was able to completely unleash himself by playing the piano, allowing himself to be fully engaged in the beautiful music. In addition, Xiao Xi gradually began to communicate with his parents in simple language, and his ability to communicate with the outside world and understand the language of others improved. Interviews with her family confirmed that an appropriate teaching method could keep the child's interest in the piano and improve her autistic condition. The author suggests that, in the future, the author can learn more about the special characteristics of this group of children by teaching them and drawing lessons through the steps of observing the problem—finding a solution—solving the problem—observing the results, and explore the appropriate teaching methods and strategies for the general teaching population in the classroom for children with autism. In the classrooms of children with autism, we have explored teaching methods and strategies that are suitable for the general teaching population and implemented and used them.

## 6. Conclusion

This study focuses on the principle and process of music intervention therapy for people with isolation disorder and designs a music regulation system based on piano performance to alleviate psychological trauma in people with psychological isolation disorder. The Emotive EPOC+ device was chosen as the EEG signal acquisition device in this study. The device is connected wirelessly via Bluetooth and is highly portable. The software system designed in this study can assist music therapists in observing and judging the emotional state of children with autism during their music therapy, solving the problem that music therapists can only switch music materials based on experience when treating children with autism. After verifying the feasibility of the algorithm, this study used the Emotive EPOC+ EEG device in the music conditioning system to acquire EEG signals from three children with autism and two adult males. A large amount of EEG signal data was successfully collected through the experiment, and three classes of positive, neutral, and negative emotion samples were completed according to the previous algorithm validation, with an average accuracy of 80.08% for the emotion recognition of the withdrawn children. Although the music regulation system based on piano performance to alleviate the psychological trauma of psychologically withdrawn people has been developed, there are still many areas for improvement, such as adding more humanized functions and combining other intervention therapies for withdrawn children with EEG technology, for example, adding VR function to increase the experience of withdrawn children during music therapy.

## Figures and Tables

**Figure 1:** Relationship between the population and the environment of autism.

**Figure 2:** Comparison of results of recognition accuracy.

**Figure 3:** Average correct rates of the experimental and control groups in different conditions.

**Figure 4:** Flowchart of the system based on piano performance to alleviate psychological trauma of people with psychological isolation disorder.

**Figure 5:** Accuracy of different parameters for identifying anxiety and calming emotions.

**Figure 6:** Sample entropy mean.

**Figure 7:** Comparison of results of self-assessment values.

**Figure 8:** Heart rate variation under different piano repertoire.

**Figure 9:** Graph of the number of emotional behaviors occurring with piano playing intervention.

## Data Availability

The data used to support the findings of this study are included within the article.
